# Integrating postpartum contraceptive counseling and IUD insertion services into maternity care in Nepal: results from stepped-wedge randomized controlled trial

**DOI:** 10.1186/s12978-019-0738-1

**Published:** 2019-05-29

**Authors:** Elina Pradhan, David Canning, Iqbal H. Shah, Mahesh Puri, Erin Pearson, Kusum Thapa, Lata Bajracharya, Manju Maharjan, Dev C. Maharjan, Lata Bajracharya, Ganga Shakya, Pushpa Chaudhary

**Affiliations:** 1 The World Bank Group, 1818 H Street NW, Washington, DC 20433 USA; 2 Department of Global Health and Population, Harvard T. H. Chan School of Public Health, 665 Huntington Avenue, Boston, MA 02115 USA; 3 Center for Research on Environment, Health and Population Activities (CREHPA), Kusunti, Lalitpur, P.O. Box 9626, Kathmandu, Nepal; 4 Ipas, P. O. Box 9990, Chapel Hill, NC 27515 USA; 5 Nepal Society of Obstetricians and Gynaecologists (NESOG), Paropakar Maternity & Women’s Hospital, Thapathali, Kathmandu, 23700 Nepal; 6 Ministry of Health and Population, Kathmandu, Nepal

**Keywords:** Nepal, Postpartum contraception, Counseling, IUD uptake, Impact evaluation

## Abstract

**Background:**

In Nepal, 54% of women have an unmet need for family planning within the 2 years following a birth. Provision of a long-acting and reversible contraceptive method at the time of birth in health facilities could improve access to postpartum family planning for women who want to space or limit their births. This paper examines the impact of an intervention that introduced postpartum contraceptive counseling in antenatal care and immediate postpartum intra-uterine device (PPIUD) insertion services following institutional delivery, with the intent to eventually integrate PPIUD counseling and insertion services as part of routine maternity care in Nepal.

**Methods:**

This study took place in six large tertiary hospitals. All women who gave birth in these hospitals in the 18-month period between September 2015 and March 2017 were asked to participate. A total of 75,587 women (99.6% consent rate) gave consent to be interviewed while in postnatal ward after delivery and before discharge from hospital. We use a stepped-wedge cluster randomized design with randomization of the intervention timing at the hospital level. The baseline data collection began prior to the intervention in all hospitals and the intervention was introduced into the hospitals in two steps, with first group of three hospitals implementing the intervention 3 months after the baseline had begun, and second group of three hospitals implementing the intervention 9 months after the baseline had begun. We estimate the overall effect using a linear regression with a wild bootstrap to estimate valid standard errors given the cluster randomized design. We also estimate the effect of being counseled on PPIUD uptake.

**Results:**

Our Intent-to-Treat analysis shows that being exposed to the intervention increased PPIUD counseling among women by 25 percentage points (pp) [95% CI: 14–40 pp], and PPIUD uptake by four percentage points [95% CI: 3–6 pp]. Our adherence-adjusted estimate shows that, on average, being counseled due to the intervention increased PPIUD uptake by about 17 percentage points [95% CI: 14–40 pp].

**Conclusions:**

The intervention increased PPIUD counseling rates and PPIUD uptake among women in the six study hospitals. If counseling had covered all women in the sample, PPIUD uptake would have been higher. Our results suggest that providing high quality counseling and insertion services generates higher demand for PPIUD services and could reduce unmet need.

**Trial registration:**

Trial registered on March 11, 2016 with ClinicalTrials.gov, NCT02718222.

## Plain English summary

Intra-uterine contraceptive device (IUD) inserted soon after delivery provides long-term protection against unintended pregnancy and can be a particularly suitable option for women who visit hospitals for delivery, but may not revisit because of distance or cost of transportation. Therefore, an intervention launched in Nepal: (1) counseled women on family planning methods after delivery during their antenatal care visits, (2) trained medical staff to insert IUD following delivery, referred as the postpartum period, and (3) thus aimed to integrate postpartum family planning, and postpartum IUD (PPIUD) services into regular maternity services. We examine the impact of this intervention on contraceptive counseling and PPIUD uptake. All women who gave birth in six tertiary hospitals in the 18-month period between September 2015 and March 2017 were asked to participate and 75,587 women who agreed were interviewed after delivery and before discharge from hospital. Baseline data were collected for 3 months in first group of hospitals after which intervention was launched in these hospitals, and the second group of hospitals had 9 months of baseline data collection before the intervention was launched. Our analysis shows that the intervention increased PPIUD counseling by 25 percentage points. It also increased PPIUD uptake by four percentage points. If all women were counseled by the program, PPIUD uptake would have increased by 17 percentage points. Our results suggest that providing high quality counseling and insertion services generates higher demand for PPIUD services and could help women meet their fertility desires to space or limit childbearing in Nepal and in similar contexts.

## Background

Increased access to family planning in low-income countries is linked to reduced maternal morbidity and mortality, and reduced infant and child morbidity and mortality [1–4]. The International Conference on Population and Development (ICPD) Programme of Action that was adopted by 179 UN member states in 1994 advocated the right to plan a family size and birth spacing as central reasons for expanding family planning access [5, 6]. Globally, although there has been an impressive increase in access to family planning in the last few decades [7], much work remains in ensuring the ICPD goals of provision of universal access to reproductive health services, including family planning.

In Nepal, contraceptive prevalence among married women aged 15–49 years increased from 19 to 53% between 1990 and 2016, and while the unmet need for family planning decreased from 34 to 24% over the same period [7, 8], concerted efforts are still needed to increase access, especially in the postpartum period. Only 9% of the women are counseled on family planning during their postpartum period in Nepal, and 54% have an unmet need for family planning within the 2 years following a birth [8]. Despite the World Health Organization’s (WHO) recommendation of waiting at least 2 years after a live birth before attempting the next pregnancy to reduce the risk of adverse maternal, perinatal and infant outcomes [9], 25% of women in Nepal become pregnant within 24 months postpartum [10]. Hence, there is a gap in postpartum family planning (PPFP) counseling and uptake in Nepal, and with rising coverage of antenatal care (ANC) and institutional delivery, an opportunity to understand whether an attempt to integrate postpartum family planning services into maternity care would improve uptake of postpartum family planning in Nepal.

Global rates of antenatal care visits and skilled birth attendance have increased in the past decades [11], and Nepal is no exception. In the period 2014–2016, 84% of women who gave birth had at least one antenatal care visit, and 57% of all births took place in a health facility (skilled birth attendance was 58%) [8]. This is a sharp increase from 2001 when only 9% of the women gave birth in a health facility in Nepal [12].

For many women in Nepal who have limited access to healthcare services, antenatal visits, facility delivery, and postnatal visits present important opportunities for counseling and provision of family planning services, which may enable them to meet their birth spacing or limiting desires by offering a long-acting and reversible method [13].

Offering family planning counseling during antenatal visits, and provision of an IUD in immediate postpartum period (PPIUD) to women undertaking delivery in a health facility can be an effective way of reducing the unmet need for family planning in the postpartum period. IUD is a safe, effective, long-lasting and reversible method of contraception [14, 15]. PPIUD, inserted in the immediate postpartum period: (1) is associated with fewer side effects and discomfort during insertion compared to an interval IUD (inserted after more than 4 weeks postpartum), (2) has higher continuation rates at 6 months [16], and (3) is recommended by the WHO as safe for use by all women, including breastfeeding women or women who are HIV positive [15].

Previously published studies on the impact of provision of PPIUD services have been based on cross-sectional and/or program data. One such recent study was a large multi-country implementation program that incorporated provision of PPIUD services into routine maternity care in six countries—Guinea, India, Ethiopia, the Philippines, Rwanda and Pakistan. This study showed that, among women counseled, between 2.3 to 5.8% chose PPIUD, and a median of about 2% of all women who gave birth in the study facilities took up PPIUD [13].

We believe this is the first study that aims to investigate the causal impact of provision of PPFP counseling and PPIUD insertion services as a part of routine maternity care. We use a randomized stepped-wedge cluster design to evaluate the causal impact of the provision of these services by employing a hospital level randomized rollout with hospitals adopting the intervention in two waves that were 6 months apart. This allows us to estimate the impact of the intervention while controlling for underlying trends in PPIUD use. The aim of this paper is to estimate the impact of the intervention on PPIUD counseling and uptake using data collected from women after delivery and before discharge from hospital—by measuring the intervention uptake, we hope to understand the feasibility of integrating PPFP counseling and PPIUD insertion services into facility-based antenatal and delivery care in Nepal.

The intervention aimed to change provider knowledge and behavior by training them on postpartum family planning, including PPIUD counseling and insertion techniques, and to change patient knowledge and behavior through counseling by the trained providers. However, human resource constraints in health facilities could attenuate the impact of the training program on PPIUD counseling and uptake [17]. Since not all women who delivered after the intervention began were counseled, we also provide adherence-adjusted estimates of the effect of being counseled on PPIUD uptake. This gives the causal effect of being counseled due to the intervention on PPIUD uptake, removing any selection bias of targeting particular women. Moreover, it has been shown that the quality of PPIUD counseling can affect uptake of PPIUD [18]. We therefore estimate how variations in the quality of counseling affected PPIUD uptake.

## Methods

This trial is registered with ClinicalTrials.gov with ID: NCT02718222. Detailed study protocol has been published elsewhere [19]. However, main features of the study are described below.

### Study population

This study took place in six tertiary hospitals: Bharatpur Hospital, Bheri Zonal Hospital, BP Koirala Institute of Health Sciences (BPKIHS), Koshi Zonal Hospital, Lumbini Zonal Hospital and Western Regional Hospital. Four of the study hospitals are in Terai region, and two (BPKIHS and Western Regional Hospital) in Hill region. Figure 1 shows a map with the location of these hospitals. The inclusion criteria for hospital sites in this study were: (i) high volume of obstetric caseloads (> 6000 a year), (ii) large catchment area, and (iii) not located in the capital city, with the intent to ascertain if the intervention could successfully build capacity in hospitals outside of Kathmandu valley. All women who gave birth in these six hospitals in the 18-month period between 8th September 2015 and 8th March 2017 were eligible to be included in the study sample unless their primary residence was outside of Nepal. Out of a total of 75,897 women eligible to enroll in the research study during the enrollment period, 75,587 (99.6%) consented to be interviewed, and interviews were conducted after delivery but prior to discharge from hospital. The full sample used in this study constitutes of 75,566 women with complete information among those who consented to participate in the study.

**Fig. 1:** Location of Study Hospitals

Ethical approval for this study was obtained through Nepal Health Research Council, and the Harvard T. H Chan School of Public Health Office of Human Research Administration granted exempt status to the study as Harvard only received de-identified data.

### Study design

We use a stepped-wedge cluster randomized design. All hospitals had at least 3 months of baseline data collection, and the intervention was introduced into the hospitals in two steps. Six hospitals were placed in pairs matched by geography (Hill versus Terai), and then by the annual obstetric caseload. Each pair was randomized into either group 1 (early intervention) or group 2 (late intervention). The three pairs were: (i) Western Regional and BPKIHS, (ii) Lumbini Zonal and Bharatpur, and (iii) Koshi Zonal and Bheri Zonal. The three hospitals in Group 1 (Lumbini Zonal, Koshi Zonal and Western Regional) were scheduled to start their intervention in the fourth month after 3-month baseline data collection, and Group 2 hospitals (BPKIHS, Bharatpur and Bheri Zonal) were scheduled to start their intervention in the tenth month after 9-month baseline data collection. Figure 2 shows the baseline and intervention period in each of the six hospitals. All hospital baseline data collection began on September 8, 2015. Actual timing of the start of the intervention by hospitals in each group varied slightly due to the need for trainers to move between hospitals to provide training. Group 1 hospitals began the intervention a few weeks apart from each other, in December 2015, whereas the intervention in Group 2 began in the summer of 2016.

**Fig. 2:** Intervention Timeline in Study Hospitals. Note: X-axis timeline is from 08 September 2015 to 08 March 2017. (1) or (2) indicates hospital group

### The intervention

The intervention was designed and implemented by International Federation of Gynecology and Obstetrics (FIGO) in partnership with Nepal Society of Obstetricians and Gynaecologists (NESOG). FIGO and NESOG designed the intervention in adherence with the national health systems and training guidelines and in coordination with the Ministry of Health and Population in Nepal to ensure sustainability of any future scale-up of the program.

The intervention comprised of: (1) informational workshops for female community health volunteers and general hospital staff, (2) training of maternity care providers in postpartum family planning counseling, PPIUD insertion techniques and complication management, (3) provision of postpartum family planning leaflets to be distributed during counseling, (4) an information wall chart and video to be displayed in the hospital waiting area, (5) provision of Kelley’s forceps for vaginal PPIUD insertion and IUDs to be provided to hospitals by the Ministry of Health and Population (IUDs were free at point-of-care to women), (6) one service provider in each hospital being designated as facility coordinator for the program, and (7) regular monitoring of counseling and insertion data by NESOG and FIGO.

#### *Provider training*

Health professionals in the study hospitals who provide obstetric services—senior and junior doctors, nurses and midwives—were trained to provide postpartum family planning counseling services during antenatal visits, and to undertake PPIUD insertions. Each training workshop was 3 days long with six sessions, which included techniques in providing counseling services along with lectures, videos, practice IUD insertion sessions in MAMA-U mannequin models for vaginal and intra-caesarian procedures, and discussion of infection prevention, side-effects and complication management. Pre-training and mid-training knowledge assessments were also conducted along with role plays and group discussions to facilitate the training.

The providers were also trained to utilize postpartum family planning leaflets during counseling. These leaflets contain information about benefits of birth spacing, and information on different contraceptives, with guidelines on when to begin using them postpartum.

#### *Counseling and consent for insertion, and intervention inclusion criteria*

If a woman in the study was counseled on PPIUD, she could have been counseled either during her antenatal visit if she visited the hospital for antenatal care (ANC), or during her postnatal care (PNC) in a ward after delivery, or in antenatal wards if she arrived early for the birth and was not in active labor. She could also be counseled both during ANC and after admission to the hospital for delivery.

If women chose to have a PPIUD inserted, consent for insertion was taken at the point of choice (either at ANC or PNC), and confirmed and noted in maternity records immediately before the insertion process. For literate women, the consent was in written form, and thumb print was taken if women were illiterate. Though the consent form was in Nepali, women were explained the process and content of the consent form in their own language by providers. Note that IUDs are provided for free at point-of-care based on national reproductive health policy guidelines, and the IUDs used in the intervention sites were non-hormonal IUDs that last 12 years.

In terms of the intervention inclusion criteria, all pregnant women who visited the hospital for antenatal counseling or delivery services (vaginal or caesarean section) were eligible for PPFP counseling services, and all those who consented to PPIUD were eligible for IUD insertion in the immediate postpartum period.

### Data collection and composition of the questionnaire

Enumerators posted in the hospitals interviewed women in the postnatal wards using structured questionnaires and the data were recorded electronically on hand-held tablets. The study questionnaire included questions about women’s socio-demographic background, birth history, ANC visits, previous contraceptive use, any family planning and PPIUD counseling received during the antenatal or postnatal period, their satisfaction with these counseling services, uptake of PPIUD, and future fertility desires.

### Outcomes of interest and key treatment variable

PPIUD counseling is a binary variable that indicates whether the woman reported receiving counseling for PPIUD either during ANC or after admission to the hospital for delivery. PPIUD uptake is also defined as an indicator variable for women who chose to accept insertion of a PPIUD. There were 27 women in our study who choose to accept PPIUD as postpartum contraception but did not receive a PPIUD because of complications during delivery and/or insertion. These women are defined as having chosen PPIUD because we intend to measure demand for PPIUD as a result of the intervention. Our key “treatment” variable is exposure to the intervention defined as delivering in a hospital after the start of the intervention as set out in Fig. 2.

### Analytic strategy

Our intention-to-treat analysis (ITT) estimates the impact of the intervention on PPIUD counseling and PPIUD uptake. This impact was analyzed using a linear regression explaining the outcome (whether counseled on PPIUD and whether PPIUD was requested) with exposure to the intervention controlling for hospital fixed effects and month fixed effects to adjust for differences between hospitals and any underlying time trends. The differential timing of the intervention across hospitals allows us to identify the effect of the intervention separately from pure time effects. We provide estimates with just these hospital-level and time dummy explanatory variables, and with additional controls for the background characteristics of the women.

While the outcome variable is binary, we have a fully saturated model with discrete explanatory variables where every individual is in one of a finite number of strata; in this case, the prediction of the outcome given by the linear probability model is simply the average outcome for the stratum, and hence is a well-specified model for the binary outcome of PPIUD uptake. We can therefore estimate the intention-to-treat effect using a simple linear regression and the treatment effect is simply the difference in outcomes between the treatment and control groups [20].

Equation 1 below represents our basic ITT model, where the dependent variable *y*_*iht*_ is a dummy variable indicating PPIUD counseling received, or PPIUD uptake, by woman i who gave birth in hospital h, on day t. The main explanatory variable of interest is *Post*_*ht*_ which is an indicator variable that takes the value one in hospital h on day t after the start of the intervention and zero before the start of the intervention. The set of *d*_*h*_ variables represents hospital fixed effects for hospitals (h) 1 through 5, with hospital 0 as reference. The set of *τ*_*m*_ variables represent month fixed-effects dummies for months 1 through 17 of the study with month 0 as reference. The *X*_*i*_ represents a vector of variables representing the characteristics of woman i. We report results with (1) only the hospital, and time fixed effects and intervention effect, and (2) additional results where we also include these additional woman level variables.

Our regression is therefore:

1 $$ {y}_{iht}=\alpha +\beta Pos{t}_{ht}+\sum \limits_{h=1}^5{d}_h+\sum \limits_{m=1}^{17}{\tau}_m+\gamma {X}_i+{\epsilon}_{iht} $$

Our primary interest is in the coefficient *β* which is the effect of the intervention. However, not all women in the intervention hospitals were counseled. Women may not have visited the study hospitals for antenatal care, receiving care at local clinics nearer their homes, and therefore may not have been exposed to the intervention. We therefore also calculate an adherence-adjusted effect of the intervention on PPIUD uptake, or the impact of being counseled due to the intervention on accepting PPIUD, calculated using an instrumental variable approach [21].

Outcomes for women who visit the same hospital are likely to be correlated with each other due to unobserved hospital level variables. Hence, inference needs to be corrected for the potential correlation in the error term across women in the same hospital. Since we only have six hospitals, or six clusters, in our study, the standard cluster robust variance estimator based on a large number of clusters may be invalid [22]. We use the wild cluster bootstrap method with six-point bootstrap weight distribution to estimate the statistical significance of the effect size for all models. This approach has been shown to have good properties with six clusters [23–25].

We also present results from a descriptive analysis on how the quality of counseling affects PPIUD uptake among women who were counseled. We look at how the provision of a PPIUD information leaflet, the opportunity to ask questions, and women’s knowledge of benefits or disadvantages of PPIUD, are related to the likelihood of accepting PPIUD.

Stata MP version 14.2 was used to perform all analyses (StataCorp LLC, College Station TX, USA).

## Results

Table 1 reports the descriptive statistics of the women level covariates used in the analysis. Column 1 shows the mean of each variable for the full sample of 75,566 women. Columns 2 and 3 show the mean of each variable for the Group 1 and Group 2 hospitals during the first 3 months of data collection, and before the intervention began in either group. With individual-level randomization of the intervention, we would expect the means of these covariates to be equal. Because we randomized at the hospital-level, and there are few hospitals, there may be systematic differences in the two populations. Column 4 reports a test of the hypothesis that the two groups of hospitals have the same mean characteristics for women during the pre-intervention period using the wild bootstrap method. We find that Group 2 hospitals tended to have women who had longer travel times to reach the hospital. However, other covariates appear to be balanced across the two groups of hospitals.

**Table 1:** Frequency and proportion of women in the first 3 months baseline period, by background and hospital group

	Full Sample	First three months			
		Group 1	Group 2	Difference^a^	
		Baseline		[Group 2- Group 1]	
				Estimate	*p*-value
Panel A					
Woman’s age					
< 20 years	10,815 (0.14)	917 (0.14)	1137 (0.15)	0.014	0.581
20–24 years	33,999 (0.45)	3061 (0.47)	3292 (0.45)	−0.022	0.512
25–29 years	21,236 (0.28)	1820 (0.28)	1941 (0.26)	− 0.015	0.561
> =30 years	9516 (0.13)	735 (0.11)	996 (0.14)	0.023	0.620
Woman’s schooling					
No schooling	6815 (0.09)	650 (0.10)	714 (0.10)	−0.003	0.973
Some primary	7637 (0.10)	694 (0.11)	734 (0.10)	−0.007	0.864
Some lower secondary	34,752 (0.46)	2886 (0.44)	3396 (0.46)	0.019	0.447
Some higher secondary	16,421 (0.22)	1368 (0.21)	1563 (0.21)	0.003	0.938
Some college	9941 (0.13)	934 (0.14)	958 (0.13)	−0.013	0.756
Time taken to travel from home to hospital					
< 2 h	39,041 (0.52)	3972 (0.61)	3564 (0.48)	−0.124	0.060
2–6 h	28,273 (0.37)	2150 (0.33)	2955 (0.40)	0.072	0.145
> =6 h	8252 (0.11)	411 (0.06)	847 (0.11)	0.052	0.055
Parity					
1	43,820 (0.58)	3771 (0.58)	4365 (0.59)	0.015	0.359
2	24,112 (0.32)	2077 (0.32)	2251 (0.31)	−0.012	0.463
3&+	7634 (0.10)	685 (0.10)	750 (0.10)	−0.003	0.915
Ethnicity					
Hill Brahmin	16,329 (0.22)	1574 (0.24)	1357 (0.18)	−0.057	0.543
Chhetri	10,693 (0.14)	831 (0.13)	1223 (0.17)	0.039	0.364
Janajaati	28,927 (0.38)	2135 (0.33)	3214 (0.44)	0.110	0.155
Madhesi	4975 (0.07)	514 (0.08)	421 (0.06)	−0.022	0.799
Dalit	11,139 (0.15)	1200 (0.18)	803 (0.11)	−0.075	0.157
Muslim	2126 (0.03)	173 (0.03)	217 (0.03)	0.003	0.910
Others	1378 (0.02)	106 (0.02)	131 (0.02)	0.002	0.838
Region					
Terai	53,459 (0.71)	3806 (0.58)	6114 (0.83)	0.247	0.596
Hill	21,419 (0.28)	2709 (0.41)	1123 (0.15)	−0.262	0.555
Mountain	688 (0.01)	18 (0.00)	129 (0.02)	0.015	0.418
Had abortion(s) before	3096 (0.04)	227 (0.03)	314 (0.04)	0.008	0.578
Male child born	40,742 (0.54)	3528 (0.54)	4063 (0.55)	0.012	0.565
Panel B					
Received Any FP counseling	21,678 (0.29)	544 (0.08)	624 (0.08)	0.001	0.971
Received PPIUD counseling	15,607 (0.21)	44 (0.01)	71 (0.01)	0.003	0.673
PPIUD uptake	1685 (0.02)	3 (0.00)	1 (0.00)	0.000	0.338
Total women	75,566	6533	7366		

^a^Significance of difference tested using wild cluster bootstrap method

Proportion of each category in parenthesis

Figure 3 shows the trends in PPIUD counseling rates in the six hospitals. During the baseline period, all hospitals had very low counseling rates and in all hospitals, there was a clear rise in counseling rates immediately after the intervention started. There is also some variability in counseling rates across the hospitals in the same group. Rates in Western Regional hospital were generally higher compared to the other hospitals. The highest monthly counseling rate achieved during the intervention period varied from 29 to 67% across the six study hospitals.

**Fig. 3:** Trends in PPIUD counseling rates. Note: Approximate intervention start-dates in group 1 and 2 hospitals shown by black and red vertical lines respectively. For exact dates of intervention, please see Fig. 2

The counseling on any method of family planning also increased (Fig. 4) following the intervention. Overall, counseling on any method increased by 23 percentage points (pp) [CI: 5.3–41.0 pp] following the intervention compared to the pre-intervention period.

**Fig. 4:** Trends in counseling rates for any FP method. Note: Approximate intervention start-dates in group 1 and 2 hospitals shown by black and red vertical lines respectively. For exact dates of intervention, please see Fig. 2

Table 2 shows the timing of PPIUD counseling, and selected measures of counseling quality. Around 39% of women were counseled in the antenatal period; 43% were counseled only after admission for delivery; and 18% were counseled both before and after admission. Among women who were counseled, only 50% reported having given an opportunity to ask questions during counseling sessions, and 58% reported receiving the postpartum family planning information leaflet. We asked women to recall benefits and some disadvantages of PPIUD and interviewers checked these responses against a list of benefits and disadvantages the counselors were trained to discuss with women. Among those counseled, 52% could recall only benefits of PPIUD, 23% could recall at least one benefit and one disadvantage, and 24% could not recall any benefits or disadvantages of the method, or could recall only disadvantages.

**Table 2:** Characteristics of PPIUD counseling and PPIUD knowledge if counseled

	n (prop.)
Timing of PPIUD counseling	
Before admission, during ANC	6124 (0.392)
After admission only	6644 (0.426)
Both	2838 (0.182)
PPIUD knowledge	
can’t recall any benefits/disadvantages, or recall disadvantages only	3775 (0.244)
recall any benefit(s) only	8071 (0.522)
recall both benefit(s) and disadvantage(s)	3617 (0.234)
Women given opportunity to ask questions	7823 (0.502)
Woman given a leaflet during counseling	9012 (0.578)
Total	15,463

Figure 5 shows results for the uptake of PPIUD, with very little uptake in any hospital during the baseline and evidence of uptake starting immediately after the intervention. There is high month-to-month variability with peaks and troughs in PPIUD uptake. However, the rise in PPIUD uptake is more pronounced after the training of providers and the start of the intervention, but shows a downward trend later.

**Fig. 5:** Trends in PPIUD Uptake. Note: Approximate intervention start-dates in group 1 and 2 hospitals shown by black and red vertical lines respectively. For exact dates of intervention, please see Fig. 2

Table 3 shows estimates of the effect of the intervention on PPIUD counseling in column 1 with the confidence interval in column 2. The estimate in column 1 controls only for hospital and month fixed effects, and we include results with additional characteristics of the women and birth as controls in column 3 with confidence intervals of these estimates given in column 4. On average, we find that the intervention increased the counseling rate by 25 pp. [95%CI: 14–40 pp]. Our effect estimate for the intervention does not depend on the inclusion of the individual women level controls, which is expected since these do not change much between the baseline and intervention periods and are unlikely to explain the increase in the outcome variable between the two periods.

**Table 3:** Intent-to-Treat Effect of the intervention on PPIUD counseling

	Dependent variable: Counseled on PPIUD			
	Est.	95% CI	Est.	95% CI
Post-treatment (Ref: Pre-treatment)	0.251**	[0.136–0.402]	0.251**	[0.142–0.400]
Woman’s age (Ref: < 20 years)				
20–24 years			0.017**	[0.002–0.036]
25–29 years			0.021**	[0.001–0.041]
> 29 years			0.012	[−0.017–0.045]
Woman’s schooling (Ref: No schooling)				
Some primary			0.028**	[0.003–0.045]
Some lower secondary			0.049***	[0.031–0.063]
Some higher secondary			0.061**	[0.029–0.093]
Some college or higher			0.058**	[0.029–0.091]
Time to travel from home to hospital (Ref: < 2 h)				
2–6 h			− 0.056**	[− 0.140 - -0.001]
> 6 h			− 0.080*	[− 0.181–0.045]
Parity (Ref: 1)				
2			0.056***	[0.036–0.077]
3 or more			0.086***	[0.056–0.113]
Ethnicity (Ref: Hill Brahmin)				
Chhetri			0.008	[−0.027–0.026]
Janajaati			−0.007	[− 0.047–0.022]
Madhesi			− 0.053**	[− 0.081 - -0.030]
Dalit			−0.013	[−0.030–0.003]
Muslim			−0.061**	[− 0.110 - -0.023]
Others			−0.008	[−0.024–0.006]
Region (Ref: Terai)				
Hill			0.0004	[−0.075–0.109]
Mountain			0.037	[−0.119–0.197]
Had an abortion before			0.015**	[0.003–0.047]
Male child born			0.002	[−0.008–0.012]
Constant	− 0.030	[− 0.178–0.098]	−0.088**	[− 0.165 - -0.005]
Observations	75,566		74,523	
R-squared	0.219		0.237	

All regression models adjusted for hospital and month fixed effects

Note: Difference from zero effect tested using wild cluster bootstrap method

*** *p* < 0.01, ** *p* < 0.05, * *p* < 0.1

While the intervention increased counseling rates overall, Table 3 shows that some subgroups of women were more likely to be counseled. Women aged 20–29 years of age and more educated women were more likely to receive PPIUD counseling. Madhesi and Muslim women were less likely to receive counseling, as were those who had long travel distances to the hospital. Counseling rates were higher among women with high parity, and among women who had previously had an abortion. The distance variable may reflect a lack of counseling in the hospital in the antenatal period and exposure to staff trained in antenatal PPIUD counseling. The other factors related to being counseled may reflect provider bias in the appropriateness of the method to certain women, or some types of women refusing counseling.

We also estimate variance inflation factor (VIF) of the adjusted model to test for multicollinearity, and find that there is some collinearity with a mean VIF of 2.16, and a VIF of 3.75 for the treatment variable in the first and the second model. We decided to keep the model structure for both models as this level of VIF is considered acceptable (< 5).

In Table 4 we report the results of a similar ITT model for the effect of the intervention on PPIUD uptake. We find the intervention increased PPIUD uptake by 4.4 pp. [95%CI: 2.8–6.4 pp]. Again, the inclusion of the women level variables has little effect on our intervention effect estimate. Uptake varies across different groups of women, but this may reflect differences in counseling rates or difference in uptake conditional on being counseled.

**Table 4:** Intent-to-Treat Effect of the intervention on PPIUD uptake

	Dependent variable: PPIUD uptake			
	Est.	95% CI	Est.	95% CI
Post-treatment (Ref: Pre-treatment)	0.044***	[0.027–0.064]	0.044***	[0.028–0.064]
Woman’s age (Ref: < 20 years)				
20–24 years			− 0.004*	[− 0.008–0.001]
25–29 years			− 0.007**	[− 0.010 - − 0.004]
> 29 years			− 0.001	[− 0.008–0.008]
Woman’s schooling (Ref: No schooling)				
Some primary			0.0004	[− 0.017–0.016]
Some lower secondary			− 0.002	[− 0.020–0.009]
Some higher secondary			− 0.003	[− 0.023–0.009]
Some college			− 0.003	[− 0.024–0.012]
Time to travel from home to hospital (Ref: < 2 h)				
2–6 h			0.0006	[−0.004–0.007]
> 6 h			−0.001	[−0.014–0.007]
Parity (Ref: 1)				
2			0.022**	[0.012–0.034]
3 or more			0.030**	[0.018–0.045]
Ethnicity (Ref: Hill Brahmin)				
Chhetri			0.003*	[0.000–0.007]
Janajaati			0.003**	[0.001–0.008]
Madhesi			− 0.002	[−0.010–0.011]
Dalit			0.0001	[−0.005–0.006]
Muslim			−0.010**	[−0.025 - -0.003]
Others			0.001	[−0.007–0.010]
Region (Ref: Terai)				
Hill			−0.001	[−0.010–0.011]
Mountain			0.0007	[−0.016–0.018]
Had an abortion before			0.011**	[0.006–0.018]
Male child born			0.003**	[0.001–0.007]
Constant	−0.005**	[−0.014 - -0.001]	− 0.013	[− 0.031–0.010]
Observations	75,566		74,523	
R-squared	0.017		0.025	

All regression models adjusted for hospital and month fixed effects

Note: Difference from null tested using wild cluster bootstrap method

*** *p* < 0.01, ** *p* < 0.05, * *p* < 0.1

The ITT estimates in Table 4 show the impact of the intervention on uptake of PPIUD. However, PPIUD counseling coverage was very incomplete even during the intervention period, and many more women might have accepted PPIUD if they had been counseled. We therefore wish to estimate the effect of being counseled on PPIUD uptake; this would give us an estimate of how successful the intervention could have been if all women had been counseled. A simple estimate of the effect of counseling on PPIUD uptake is likely to be biased if counseling was targeted by providers to focus on women more likely to accept PPIUD. Indeed, in Table 3 we see that counseling is correlated with the characteristics of women that suggests some targeting of counseling may be occurring. If this is the case, extending counseling to additional women may have lower impact than in those already being counseled.

In order to avoid this problem of targeted counseling we estimate the “adherence-adjusted” effect of the intervention, the effect of the intervention on PPIUD among those counseled due purely to the intervention and not targeting. Formally, this is an instrumental variable estimate where we use the predicted probability of counseling from column 3 of Table 3 as the explanatory variable in a two-stage procedure [21]. The results in Table 5 show the effect of counseling on PPIUD uptake using this approach to remove the effect of targeting. The adherence-adjusted estimate implies that receiving counseling due to the intervention increases uptake of PPIUD by around 17 percentage points [95% CI: 14–40 pp].

**Table 5:** Adherence-adjusted Impact of the Intervention—Impact of PPIUD counseling on PPIUD uptake

	Dependent variable: PPIUD uptake			
	Est.	95% CI	Est.	95% CI
Counseled on PPIUD	0.173***	[0.098–0.246]	0.174***	[0.099–0.249]
Woman’s age (Ref: < 20)				
20–24 years			− 0.006**	[− 0.012 - -0.001]
25–29 years			− 0.009**	[− 0.014 - -0.004]
> 29 years			− 0.002	[− 0.012–0.007]
Woman’s schooling (Ref: No schooling)				
Some primary			− 0.004	[− 0.014–0.011]
Some lower secondary			− 0.009*	[− 0.023–0.001]
Some higher secondary			− 0.013**	[− 0.027 - -0.004]
Some college			− 0.013**	[− 0.028 - -0.003]
Time to travel from home to hospital (Ref: < 2 h)				
2–6 h			0.010**	[0.001–0.022]
> 6 h			0.012**	[0.005–0.019]
Parity (Ref: 1)				
2			0.013**	[0.004–0.021]
3 or more			0.016**	[0.003–0.029]
Ethnicity (Ref: Hill Brahmin)				
Chhetri			0.003	[− 0.003–0.011]
Janajaati			0.005*	[0.000–0.013]
Madhesi			0.007	[− 0.002–0.018]
Dalit			0.002	[−0.003–0.007]
Muslim			0.0003	[−0.006–0.009]
Others			0.004	[−0.007–0.020]
Region (Ref: Terai)				
Hill			−0.001	[−0.007–0.001]
Mountain			−0.007	[− 0.032–0.019]
Had an abortion before			0.010**	[0.005–0.018]
Male child born			0.002***	[0.001–0.004]
Constant	−0.0006	[−0.023–0.023]	−0.0003	[− 0.024–0.024]
Observations	75,566		74,525	
R-squared	0.053		0.058	

All regression models adjusted for hospital and month fixed effects

Note: Difference from null tested using wild cluster bootstrap method. Second Stage Results Shown. First Stage results in Table 3, Columns (1) and (2)

*** *p* < 0.01, ** *p* < 0.05, * *p* < 0.1

Table 6 shows the determinants of PPIUD uptake among women who were counseled. Women who were counseled in the hospital after admission for delivery were more likely to take up PPIUD. Our measures of the quality of counseling, in the form of having the opportunity to ask questions during counseling, and being able to remember benefits and disadvantages of PPIUD are correlated with a higher rate of PPIUD uptake. Being given a PPIUD information leaflet, however, did not seem to be related to uptake. Women with secondary or higher education are less likely to take up PPIUD, and Muslim women were less likely to choose PPIUD compared to Hill Brahmin women. PPIUD uptake was higher among women with more children, and those who wanted to space or limit their future pregnancies.

**Table 6:** Determinants of PPIUD uptake among women who were counseled

	Dependent variable: PPIUD uptake	
	Est.	95% CI
Woman given a leaflet during counseling	−0.008	[− 0.050–0.053]
PPIUD Knowledge (Ref: Women can’t recall any benefits/disadvantages, or disadvantages only)		
recall benefit(s) only	0.054**	[0.026–0.080]
recall both benefit(s) and disadvantage(s)	0.122***	[0.091–0.198]
Women given opportunity to ask questions	0.043**	[0.012–0.095]
Timing of PPIUD Counseling (Ref: Before Admission, during ANC)		
After Admission Only	0.144**	[0.096–0.237]
Both	0.093**	[0.055–0.187]
Woman’s Age (Ref: < 20)		
20–24 years	−0.020**	[−0.036–0.000]
25–29 years	−0.036**	[− 0.045 - -0.027]
> 29 years	− 0.015	[− 0.035–0.037]
Woman’s Schooling (Ref: No schooling)		
Some Primary	−0.015	[− 0.054–0.070]
Some Lower Secondary	−0.042	[− 0.072–0.013]
Some Higher Secondary	−0.045	[− 0.072–0.011]
Some College	−0.051*	[− 0.083–0.012]
Time to travel from home to hospital (Ref: < 2 h)		
2–6 h	0.008	[− 0.011–0.038]
> 6 h	− 0.0027	[−0.046–0.074]
Parity (Ref: 1)		
2	0.039**	[0.011–0.055]
3 or more	0.050*	[−0.003–0.076]
Ethnicity (Ref: Hill Brahmin)		
Chhetri	0.007	[−0.010–0.029]
Janajaati	0.010	[−0.004–0.036]
Madhesi	−0.003	[− 0.041–0.107]
Dalit	−0.002	[− 0.026–0.034]
Muslim	−0.035*	[− 0.061–0.003]
Others	0.003	[− 0.042–0.048]
Region (Ref: Terai)		
Hill	−0.008	[− 0.057–0.049]
Mountain	0.017	[− 0.145–0.144]
Had an abortion before	0.025*	[−0.006–0.042]
Male child born	0.014***	[0.006–0.027]
Future Fertility Preference (Ref: Unsure about Limiting)		
Want to Space	0.023**	[0.006–0.054]
Want to Limit	0.020***	[0.006–0.049]
Undecided on Spacing	−0.006	[−0.060–0.017]
Can’t get Pregnant	−0.119**	[− 0.240 - -0.053]
Refused/Other	−0.068**	[− 0.182 - -0.003]
Constant	−0.181	[− 0.379–0.021]
Observations	15,241	
R-squared	0.132	

All regression models adjusted for hospital and month fixed effects

Note: Difference from null tested using wild cluster bootstrap method

*** *p* < 0.01, ** *p* < 0.05, * *p* < 0.1

## Discussion

The results from this study show that the intervention had a statistically significant impact on increasing PPIUD counseling rates and PPIUD uptake among women in the six study hospitals. We further find that the impact of the intervention on PPIUD uptake was about four times larger in women who were counseled.

However, we find that only a quarter of women were counseled on family planning, and furthermore, nearly one-third of those counseled were told of only one contraceptive method. In addition, a substantial number of women were only counseled after admission to the hospital for delivery, rather than in the antenatal period. The intervention focused on training in the hospital delivery wards and their antenatal care facilities and many women, particularly those living far from a hospital, may have had their antenatal care elsewhere. There is substantial variation in counseling rates between different groups of women which may reflect access to hospital-based antenatal services but which may also reflect provider bias in the appropriateness of the method for different groups.

Quality of care is a critical factor that determines service uptake and method continuation. We found that patients who were likely offered higher quality care (women counseled on both benefits and disadvantages of the method) were more likely to take up PPIUD as compared to women offered lower quality care (women who only knew benefits or disadvantages). A paper that examined adverse effects of PPIUD insertion across six countries where this intervention was implemented found 22% of women with PPIUD reporting at least one adverse effect at 6-week follow-up, with 6.9% reporting vaginal discharge, 4.4% abdominal pain, and 2.4% irregular bleeding [26]. The same study reported expulsion rate of 3.9% by 6 weeks since PPIUD insertion in Nepal, as compared to a minimum of 1.2% in Tanzania and 4.3% in Kenya, and a removal rate of 7.4% in Nepal as compared to 2.6% in Kenya and 8.3% in Tanzania. Note that for the study above, the 6-week follow-up rate for Nepal was the highest at 84%, and was between (42–54) % for the remaining five countries indicating that the expulsion and removal data were more complete for Nepal than for the other countries. The high removal rate by women in Nepal suggests a need for improvement in quality of counseling. This may also reflect dynamics of an economy based on large number of Nepalese men working abroad where women often decide on contraceptive methods alone, and husbands, when they come back for short periods of time are not satisfied with the method as they do not receive any information or counseling on the method. These results suggest a need for modified counseling approach in Nepal catered to country-specific labor and household power dynamics.

Another aspect of quality of care is the health system readiness and provider’s capacity to deliver care. A paper examining provider perspectives on the FIGO-NESOG intervention in Nepal finds that the providers in the study hospitals were positive about implementing PPFP counseling and PPIUD insertion services as a part of routine maternity care, but identified several supply-side issues preventing them from providing high-quality care including: (1) shortage of human resources, (2) lack of supplies and (3) lack of support from the hospital management [27]. Hence, improvements in health systems readiness to deliver these services would not only improve provider morale, but could also improve counseling rates and method uptake.

Among those counseled, women who expressed their desire to limit or space their future pregnancies were more likely to take up PPIUD compared to women who were unsure about limiting. As older women and women with higher parity are more likely to want to space or limit their future pregnancies [28], higher PPIUD uptake by older women, women with high parity births, or history of abortion might mean that the intervention enabled women to meet their unmet need for family planning. This heterogeneity implies that these sub-populations might be prioritized by policymakers during scale-up to reach populations with the highest demand for postpartum contraception.

The main analytical strategy of the study was to examine the intent-to-treat effect, and the impact on those who were actually treated (that is, who were counseled). However, there is also some heterogeneity in fidelity to the intervention across the different hospital sites, where counseling rates at some hospitals in some months were as high as 67%. Examining key factors behind this heterogeneous uptake of the intervention at the hospital and even at the provider level is an important area of future research.

The women in our study are not nationally representative. On average, they are younger and have more years of schooling than women of reproductive age in Nepal [8]. In targeting tertiary hospitals with high obstetric caseloads, our study excludes women who delivered at home, or in smaller primary health care centers. The implementation design also does not include adolescent girls who also have a high unmet need for contraception primarily to delay age at first childbirth [29, 30]. By design, the study was implemented in large tertiary hospitals but in many rural areas, births either take place in lower level district hospitals, primary health centers or health posts, and it is unclear if the intervention could be implemented in these smaller facilities. Implications on program resources including costs and logistics to expand PPFP and PPIUD services to the numerous district hospitals, and other health facilities need to be weighed against the benefits of expanded reach to women who often have even more limited access to postpartum family planning, and might benefit more from a long-acting and reversible method given higher time, cost and distance barriers to seeking care from health facilities.

High unmet need of postpartum family planning, and contraceptive prevalence rate that has only moved from 48 to 52.6% in the last decade (2006 to 2016) requires that the public health system in Nepal be introduced to innovative reproductive health interventions to ensure universal access to high-quality reproductive and sexual health services. This study aimed to understand the feasibility of one such innovation, which was the attempt to integrate postpartum family planning counseling and PPIUD insertion service provision into routine maternity care services in Nepal. Our evaluation demonstrates that incorporating PPIUD services into routine maternity care is feasible, and there is a demand for the PPIUD from women who have need for spacing or limiting their births. The intervention had a reasonable impact on PPIUD counseling rates, though it fell well short of full coverage of women delivering in the intervention hospitals, and a smaller, but statistically significant impact on PPIUD uptake, particularly among those who received high-quality counseling. We conclude that the intervention had a positive impact though its effectiveness might be improved by expanding the coverage of counseling and ensuring that the counseling is of high quality.

## Conclusions

The intervention designed and implemented by FIGO and NESOG increased PPIUD counseling rates and PPIUD uptake among women, especially among older women, those with high parity, and those who received better quality counseling. Had the counseling covered all women who gave birth, PPIUD uptake would have been four times higher. Our results suggest that the program impact could be improved further by: (1) expanding the coverage of PPFP counseling during antenatal care, and (2) improving quality of counseling. Increasing the coverage of high-quality counseling will likely require increased human resources for health and a shift in emphasis to counseling during the antenatal period in health centers providing antenatal care and not just in hospital antenatal clinics.

## Abbreviations

ANC: Antenatal Care
BPKIHS: BP Koirala Institute of Health Sciences
CI: Confidence Interval
FIGO: International Federation of Obstetricians and Gynaecologists
ICPD: International Conference on Population and Development
ITT: Intention-To-Treat
IUD: Intra-Uterine Device
NESOG: Nepal Society of Obstetricians and Gynaecologists
PNC: Postnatal Care
PP: Percentage Point
PPIUD: Postpartum Intra-Uterine Device
VIF: Variance Inflation Factor
WHO: World Health Organization
